The article "Changes of Serum Ferritin, Hemoglobin, and Serum Iron (SI) and Treatment Effect of Iron Proteinsuccinylate Oral Solution Combined with Vitamin A and D Drops on Children with Nutritional Iron Deficiency Anemia" was retracted in 2024. Reasons: suspected computer-generated content; unreliable results or conclusions; concerns about the data; concerns about the results or conclusions.

# Changes of Serum Ferritin, Hemoglobin, and Serum Iron (SI) and Treatment Effect of Iron Proteinsuccinylate Oral Solution Combined with Vitamin A and D Drops on Children with Nutritional Iron Deficiency Anemia

**DOI:** 10.1155/2022/2972617

**Published:** 2022-01-13

**Authors:** Yan Ma, Yanbo Ma, Xiuqing Zhang, Xuejing Wang, Zhigang Sun

**Affiliations:** ^1^Pediatric Internal Medicine, The Second People's Hospital of Liaocheng, The Second Hospital of Liaocheng Affiliated to Shandong First Medical University, 252600 Liaocheng, Shandong Province, China; ^2^Child Healthcare Department, The Second People's Hospital of Liaocheng, The Second Hospital of Liaocheng Affiliated to Shandong First Medical University, 252600 Liaocheng, Shandong Province, China

## Abstract

**Objective:**

The purpose was to evaluate the treatment effect of iron proteinsuccinylate oral solution combined with vitamin A and D drops on children with nutritional iron deficiency anemia.

**Methods:**

124 children treated in the outpatient department of our hospital from January 2017 to January 2020 were selected as the study subjects. They were randomly divided into control and observation two groups. The control group was treated with iron proteinsuccinylate oral solution (1.5 mL/kg) in the morning and evening, respectively. The observation group received adjuvant treatment with oral vitamin A and D drops based on the treatment of the control group. The treatment effect of proteinsuccinylate oral solution combined with vitamin A and D drops was evaluated by the serum iron (SI), serum ferritin (SF), and transferrin (TRF) levels, the values of CD3^+^, CD4^+^, and CD4^+^/CD8^+^, and other evaluation indicators.

**Results:**

After treatment, the SI and SF levels of children in both groups significantly increased (*P* < 0.01) while the TRF level significantly decreased (*P* < 0.01), and the SI and SF levels in the observation group increased more significantly, and the TRF level decreased more significantly compared with those in the control group (*P* < 0.01). After treatment, the values of CD3^+^, CD4^+^, and CD4^+^/CD8^+^ of children in both groups significantly increased compared with those before treatment (*P* < 0.01), and the values of CD3^+^, CD4^+^, and CD4^+^/CD8^+^ increased more significantly in the observation group compared with those in the control group (*P* < 0.01). In addition, the evaluation results of treatment effect showed that the markedly effective rate in the observation group was significantly higher than that in the control group (*P* < 0.01).

**Conclusion:**

Iron proteinsuccinylate oral solution combined with vitamin A and D drops can better improve the anemia symptoms in children, with high application value.

The article "Changes of Serum Ferritin, Hemoglobin, and Serum Iron (SI) and Treatment Effect of Iron Proteinsuccinylate Oral Solution Combined with Vitamin A and D Drops on Children with Nutritional Iron Deficiency Anemia" was retracted in 2024. Reasons: suspected computer-generated content; unreliable results or conclusions; concerns about the data; concerns about the results or conclusions.

## 1. Introduction

Iron, an essential trace element in human body, plays an important role in maintaining the activities of hemoglobin, myoglobin, and metabolic-related enzymes in human body and can participate in various physiological activities of human body. Patients with iron deficiency are often accompanied by oxygen transport disorders, resulting in metabolic disorders and eventually anemia [1–3]. Iron deficiency anemia is more common in children, whose pathogenesis has a variety of reasons including unreasonable dietary structure, massive iron loss caused by chronic bleeding, and iron malabsorption in the body, which has a serious impact on the development and growth of children [4–6]. At present, to treat this chronic disease, dietary therapy, iron preparations, and other methods are often used in the intervention, including increasing the intake of liver, lean meat, and soy products to improve the internal environment of children or directly supplementing iron preparations to raise the iron level in the body, promoting the synthesis of hemoglobin in vivo and thereby improve the symptoms of anemia [7–9]. In clinic, iron preparations for the treatment of iron deficiency anemia in children mainly include ferrous gluconate and iron proteinsuccinylate [10–12]. However, some studies have shown that iron deficiency anemia is associated with some vitamin deficiencies in children [13, 14]. Based on this, 124 children treated in the outpatient department of our hospital from January 2017 to January 2020 were selected as the study subjects in this study. Vitamin A and D drops were used based on iron proteinsuccinylate to evaluate the symptom improvement before and after treatment through SI, SF, TRF, and immune levels, which is aimed at providing a reference for the treatment of iron deficiency anemia in children.

## 2. Materials and Methods

### 2.1. General Information

This study was approved by the hospital ethics committee. 124 children treated in the outpatient department of our hospital from January 2017 to January 2020 were selected as the study subjects. The general data of the patients are shown in Table 1.

### 2.2. Screening Criteria

Inclusion criteria are as follows: (1) the patients were clinically diagnosed with iron deficiency anemia; (2) the guardians of the children had a detailed understanding of the content of the study; (3) the patient had symptoms such as pale skin, decreased appetite, and depression; (4) the guardians of the children voluntarily signed the informed consent; (5) the children were aged 3-9 years old; (6) the children had never received intervention with iron preparations.

The article "Changes of Serum Ferritin, Hemoglobin, and Serum Iron (SI) and Treatment Effect of Iron Proteinsuccinylate Oral Solution Combined with Vitamin A and D Drops on Children with Nutritional Iron Deficiency Anemia" was retracted in 2024. Reasons: suspected computer-generated content; unreliable results or conclusions; concerns about the data; concerns about the results or conclusions.

Exclusion criteria are as follows: (1) children with hemolytic anemia, (2) children with aplastic anemia, (3) children with iron utilization disorder and other symptoms, (4) children with hematopoietic disorder, and (5) children could not cooperate with clinical follow-up.

### 2.3. Treatment Methods

124 children were randomly divided into two groups for control and observation. The children in the control group were treated with iron proteinsuccinylate oral solution, once in the morning and once in the evening, with a total dose of 1.5 mL/kg. The children in the observation group received adjuvant treatment with vitamin A and D drops based on the treatment of the control group, with oral administration of one vitamin A (12,000 IU/pill) and one vitamin D_3_ (700 IU/pill) daily.

Drug information is as follows: iron proteinsuccinylate oral solution (Italfarmaco S.p.A; SFDA No.: H20160143) and vitamin A and D drops (Shandong Dyne Marine Biopharmaceutical Co., Ltd.; SFDA No.: H37022974).

### 2.4. Observation Indexes

*Determination of SI, SF, and TRF levels*: 2 mL of venous blood was taken before and after treatment in fasting state to detect SI, SF, and TRF levels. Bipyridine colorimetry was used to detect the SI, and chemiluminescence immunoassay was used to detect the SF and TRF levels.

*Determination of immune level*: the levels of CD3^+^, CD4^+^, and CD8^+^ of T lymphocyte subsets in children were measured by a flow cytometry, and the ratio of CD4^+^/CD8^+^ was calculated.

*Clinical efficacy*: the treatment effect was divided into markedly effective, effective, and ineffective according to the appetite, spirit, skin, and mucosal color of children, SI, SF, and TRF levels, and the improvement of CD3^+^, CD4^+^, and CD4^+^/CD8^+^ of children.

### 2.5. Data Analysis

The data obtained in this study were processed by SPSS 20.0. The measurement data and count data were tested by *t*-test and *χ*^2^, respectively. The difference was statistically significant when *P* < 0.05.

## 3. Results

### 3.1. Comparison of SI Levels between the Two Groups of Children before and after Treatment

The SI levels of children in the two groups before and after treatment are shown in Figure 1. After treatment, the SI levels of children in both groups significantly increased compared with those before treatment (*P* < 0.01), and the SI level in the observation group increased more significantly compared with that in the control group (*P* < 0.01).

### 3.2. Comparison of SF Levels between the Two Groups of Children before and after Treatment

The SF levels of children in the two groups before and after treatment are shown in Figure 2. After treatment, the SF levels of children in both groups significantly increased compared with those before treatment (*P* < 0.01), and the SF level in the observation group increased more significantly compared with that in the control group (*P* < 0.01).

The article "Changes of Serum Ferritin, Hemoglobin, and Serum Iron (SI) and Treatment Effect of Iron Proteinsuccinylate Oral Solution Combined with Vitamin A and D Drops on Children with Nutritional Iron Deficiency Anemia" was retracted in 2024. Reasons: suspected computer-generated content; unreliable results or conclusions; concerns about the data; concerns about the results or conclusions.

### 3.3. Comparison of TRF Levels between the Two Groups of Children before and after Treatment

The serum TRF levels of children in the two groups before and after treatment are shown in Figure 3. After treatment, the serum TRF levels of children in both groups significantly decreased compared with those before treatment (*P* < 0.01), and the TRF level in the observation group decreased more significantly compared with that in the control group (*P* < 0.01).

### 3.4. Comparison of the Immune Level between the Two Groups of Children before and after Treatment

The changes of immune level of children in the two groups before and after treatment are shown in Table 2. After treatment, the values of CD3^+^, CD4^+^, and CD4^+^/CD8^+^ of children in both groups significantly increased compared with those before treatment (*P* < 0.01), and the values of CD3^+^, CD4^+^, and CD4^+^/CD8^+^ increased more significantly in the observation group compared with that in the control group (*P* < 0.01).

### 3.5. Comparison of Treatment Effect between the Two Methods

The treatment effect of the two methods is shown in Table 3. The proportion of children with obviously improved symptoms in the observation group was significantly higher than that in the control group (*P* < 0.05).

## 4. Discussion

Iron deficiency anemia is a common chronic disease in children, which not only leads to poor body development and slow growth of children but also seriously affects their intellectual development [15, 16]. Iron proteinsuccinylate is a widely used iron supplement in clinical practice, which can effectively improve the iron deficiency in children. However, iron deficiency anemia in children is a comprehensive metabolic disease, and the treatment of simply supplementing iron has certain limitations [17, 18]. Therefore, it is of positive significance to select a reasonable treatment for children with iron deficiency anemia.

SI, SF, and TRF levels are often used to reflect the severity of iron deficiency anemia in patients [19]. In this study, the changes of SI, SF, and TRF levels of children were used to reflect their iron level in vivo. Compared with those before treatment, the SI and SF levels of children in both groups increased significantly after treatment while the TRF level decreased significantly, indicating that long-term administration of iron proteinsuccinylate could significantly improve the body iron level of children and thereby improve the symptoms of anemia. Iron proteinsuccinylate is a commonly used iron supplement in clinical practice, which is often used to treat anemia caused by iron malabsorption in pregnant and lactating women and children. In addition, compared with the control group, the SI and SF levels of children in the observation group increased more significantly after treatment while the TRF level decreased more significantly, indicating that the adjuvant treatment of vitamin A and D drops can better improve the iron deficiency in children, so as to further alleviate the anemia symptoms. The vitamin A level is significantly correlated with iron deficiency anemia in children. Larson et al. [20] found that vitamin A could directly reflect the degree of anemia in preschool and school-age children as an independent factor through investigation. In addition, Altemose et al. [21] showed that vitamin D deficiency also increased the risk of iron deficiency anemia in children. These studies indicate that increased vitamins A and D can help improve the symptoms of anemia in children.

The article "Changes of Serum Ferritin, Hemoglobin, and Serum Iron (SI) and Treatment Effect of Iron Proteinsuccinylate Oral Solution Combined with Vitamin A and D Drops on Children with Nutritional Iron Deficiency Anemia" was retracted in 2024. Reasons: suspected computer-generated content; unreliable results or conclusions; concerns about the data; concerns about the results or conclusions.

The immune level of children is significantly correlated with the content of iron ions in their blood and can directly reflect their health [22]. In this study, the levels of CD3^+^ and CD4^+^ and the ratio of CD4/CD8 were used to observe the changes in immunity of children before and after treatment. Compared with those before treatment, the levels of CD3^+^ and CD4^+^ and the ratio of CD4/CD8 in both groups increased significantly after treatment, indicating that long-term administration of iron proteinsuccinylate can significantly improve the immunity of children, thereby effectively reducing the incidence of complications caused by iron deficiency anemia in children. In addition, compared with the control group, the levels of CD3^+^ and CD4^+^ and the ratio of CD4/CD8 increased more significantly in the observation group after the adjuvant treatment of vitamin A and D drops, indicating that vitamin A and D drops as an adjuvant treatment could better improve the immunity of children and effectively improve their health level. Studies have shown that the deficiency of vitamins A and D is significantly related to the incidence of various diseases in children, and the supplementation of vitamins A and D can effectively improve the immune level of children and enhance their resistance to viruses [23, 24]. These studies suggest that vitamin A and D supplementation can help to improve the immune level of children. In addition, Houghton et al. [25] found that the majority of children with iron deficiency anemia included in their study had severe deficiencies in vitamins A and D. This finding also supports the conclusion of this study, indicating that vitamin A and D supplementation has a positive effect on improving the symptoms of anemia in children.

The article "Changes of Serum Ferritin, Hemoglobin, and Serum Iron (SI) and Treatment Effect of Iron Proteinsuccinylate Oral Solution Combined with Vitamin A and D Drops on Children with Nutritional Iron Deficiency Anemia" was retracted in 2024. Reasons: suspected computer-generated content; unreliable results or conclusions; concerns about the data; concerns about the results or conclusions.

In conclusion, our study demonstrated that iron proteinsuccinylate oral solution combined with vitamin A and D drops can better improve the anemia symptoms in children, indicating this approach can transform nutritional status assessment and monitoring globally.

## Figures and Tables

**Figure 1:** Comparison of SI levels between the two groups of children before and after treatment. Note: The abscissa represents the groups, and the ordinate represents the SI level of patients. ∗ indicated that there was a significant difference in the SI levels of children in the control group before treatment (11.97 ± 2.13 *μ*mol/L) and after treatment (15.09 ± 3.69 *μ*mol/L; *t* = 4.99 and *P* = 1.6*e* − 5). ∗∗ indicated that there was a significant difference in the SI levels of children in the observation group before treatment (11.99 ± 2.09 *μ*mol/L) and after treatment (16.91 ± 3.71 *μ*mol/L; *t* = 4.50 and *P* = 8.2*e* − 5). ∗∗∗ indicated that there was a significant difference in the SI levels of children in both groups after treatment (*t* = 2.74 and *P* = 4.5*e* − 3).

**Figure 2:** Comparison of SF levels between the two groups of children before and after treatment. Note: The abscissa represents the groups, and the ordinate represents the SF level of patients. ∗ indicated that there was a significant difference in the SF levels of children in the control group before treatment (85.31 ± 8.96 *μ*g/L) and after treatment (156.19 ± 12.97 *μ*g/L; *t* = 3.84 and *P* < 0.01). ∗∗ indicated that there was a significant difference in the SF levels of children in the observation group before treatment (85.69 ± 8.99 *μ*g/L) and after treatment (173.32 ± 13.32 *μ*g/L; *t* = 3.47 and *P* < 0.01). ∗∗∗ indicated that there was a significant difference in the SF levels of children in both groups after treatment (*t* = 7.26 and *P* < 0.01).

**Figure 3:** Comparison of TRF levels between the two groups of children before and after treatment. Note: The abscissa represents the groups, and the ordinate represents the serum TRF level of patients. ∗ indicated that there was a significant difference in the serum TRF levels of children in the control group before treatment (7.23 ± 1.21 *μ*g/L) and after treatment (3.77 ± 0.61 *μ*g/L; *t* = 12.41 and *P* < 0.01). ∗∗ indicated that there was a significant difference in the serum TRF levels of children in the observation group before treatment (7.29 ± 1.09 *μ*g/L) and after treatment (2.95 ± 0.43 *μ*g/L; *t* = 16.38 and *P* < 0.01). ∗∗∗ indicated that there was a significant difference in the serum TRF levels of children in both groups after treatment (*t* = 8.65 and *P* < 0.01).

The article "Changes of Serum Ferritin, Hemoglobin, and Serum Iron (SI) and Treatment Effect of Iron Proteinsuccinylate Oral Solution Combined with Vitamin A and D Drops on Children with Nutritional Iron Deficiency Anemia" was retracted in 2024. Reasons: suspected computer-generated content; unreliable results or conclusions; concerns about the data; concerns about the results or conclusions.

**Table 1:** General information of patients.

Items	Control group	Observation group	*t*	*P*
Sex ratio	15 : 16	1 : 1	0.03	0.83
Average age (years old)	6.73 ± 0.53	6.69 ± 0.59	0.40	0.44
Body mass index (kg/m^2^)	13.98 ± 0.53	13.97 ± 0.56	0.10	0.75
SI level (*μ*mol/L)	11.98 ± 2.09	12.01 ± 2.13	0.08	0.77
SF level (*μ*g/L)	85.29 ± 8.03	85.29 ± 8.03	0.06	0.81
Serum TRF level (*μ*g/L)	7.23 ± 1.19	7.27 ± 1.11	0.19	0.63
CD3^+^ level (%)	40.29 ± 3.29	40.31 ± 3.27	0.03	0.83
CD4^+^level (%)	37.09 ± 2.09	37.03 ± 2.07	0.16	0.71

**Table 2:** Immune level of children in two groups.

Indicators	Groups	Cases	Before treatment	After treatment	*t*	*P*
CD3^+^ (%)	Control group	62	40.32 ± 3.57	49.13 ± 3.35	5.88	6.5*e*-6
	Observation group	62	40.27 ± 3.16	55.09 ± 4.19	5.29	3.1*e*-6
	*t*		0.08	8.75		
	*P*		0.77	5.6*e*-8		

CD4^+^ (%)	Control group	62	37.13 ± 2.21	41.97 ± 3.03	6.53	9.6*e*-7
	Observation group	62	37.29 ± 2.13	45.29 ± 3.31	6.10	3.6*e*-7
	*t*		0.41	5.83		
	*P*		0.42	5.3*e*-6		

CD4^+^/CD8^+^	Control group	62	1.17 ± 0.19	1.39 ± 0.23	5.48	5.9*e*-6
	Observation group	62	1.15 ± 0.17	1.63 ± 0.27	4.67	5.7*e*-5
	*t*		0.62	5.33		
	*P*		0.31	4.9*e*-6		

**Table 3:** Treatment effect between the two methods.

Groups	Cases	Marked effective	Effective	Ineffective	Effective rate (%)
Control group	62	25	26	11	82.56
Observation group	62	36	23	3	95.16
*χ* ^2^	6.74				
*P*	0.007				

## Data Availability

The authors confirm that the data supporting the findings of this study are available within the article.
